# The *MTHFR* promoter hypermethylation pattern associated with the A1298C polymorphism influences lipid parameters and glycemic control in diabetic patients

**DOI:** 10.1186/s13098-019-0399-9

**Published:** 2019-01-15

**Authors:** Herlanny Santana Bezerra, Caroline Severo de Assis, Mayara Karla dos Santos Nunes, Isabella Wanderley de Queiroga Evangelista, João Modesto Filho, Cecília Neta Alves Pegado Gomes, Rayner Anderson Ferreira do Nascimento, Rafaella Cristhine Pordeus Luna, Maria José de Carvalho Costa, Naila Francis Paulo de Oliveira, Darlene Camati Persuhn

**Affiliations:** 1 Scientific Initiation Program, Federal University of Paraiba, Joao Pessoa, Brazil; 2 Nutrition Sciences, Federal University of Paraiba, Joao Pessoa, Brazil; 3 Development and Technological Innovation of Medicines, Federal University of Paraiba, João Pessoa, Brazil; 4 Unidade da Visão, Hospital Universitário Lauro Wanderley, Federal University of Paraíba, Joao Pessoa, Brazil; 5 Department of Internal Medicine, Federal University of Paraiba, Joao Pessoa, Brazil; 6 Nephrology Clinic, Lauro Wanderley University Hospital, Federal University of Paraiba, Joao Pessoa, Brazil; 7 Faculty Mauricio of Nassau, Joao Pessoa, Brazil; 8 Post-Graduate Program in Nutrition Science, Federal University of Paraiba, Joao Pessoa, Brazil; 9 Nutrition Science Department and Post-Graduate Program in Nutrition Science, Federal University of Paraiba, Joao Pessoa, Brazil; 10 Department of Molecular Biology, Federal University of Paraiba, Joao Pessoa, Brazil; 11 Department of Molecular Biology and Post-Graduate Program in Nutrition Science, Federal University of Paraiba, João Pessoa, PB CEP 58051-900 Brazil

**Keywords:** Methylation of DNA, Type 2 diabetes mellitus, Biochemical profile

## Abstract

**Background:**

Polymorphisms in the gene encoding methylenetetrahydrofolate reductase (MTHFR) have been investigated as risk factors for microvascular complications of diabetes; however, simultaneous analysis of these polymorphisms and the methylation pattern of the gene has never been conducted. The objective of the present study was to evaluate the simultaneous relationship between *MTHFR* methylation and *MTHFR* C6TT7 and A1298C polymorphisms with metabolic, inflammatory and oxidative stress parameters related to microvascular complications, diabetic retinopathy (DR) and diabetic nephropathy (DN) in diabetic patients.

**Methods:**

A total of 107 patients who were diagnosed in the previous 5 to 10 years were recruited and divided into groups with complications (DR and/or DN) or without complications. Methylation analysis of the gene promoter was conducted using the MSP technique, and analysis of the A1298C and C677T polymorphisms was conducted using the restriction fragment length polymorphism (RFLP) assay. Microalbuminuria was determined using urine samples, and other analytes of interest were determined in blood samples using commercial kits. The Mann–Whitney and Chi square statistical tests were used with significance considered at p < 0.05.

**Results:**

Subjects with a hypermethylated profile and the 1298AA genotype showed the highest levels of blood glucose (p = 0.03), total cholesterol (p = 0.0001) and LDL cholesterol (p = 0.0006). The same profile was associated with higher levels of HbA1c (p = 0.025), glycemia (p = 0.04) and total cholesterol (0.004) in the control group and total cholesterol (p = 0.005) and LDL cholesterol (p = 0.002) in the complications group. Serum creatinine was higher in subjects in the hypermethylated group with the genotype 677CC only in the control group (p = 0.0020). The methylated profile in presence of 677CC + 1298AA and the 677CT/TT +1298AA haplotypes showed higher levels of total cholesterol (p = 0.0024; 0.0031) and LDL cholesterol (p = 0.0060; 0.0125) than 1298AC/CC carriers. The fasting glycemia was higher in hypermethylated profile in the presence of 677CC/1298AA haplotype (p = 0.0077).

**Conclusion:**

The hypermethylated methylation profile associated with the 1298AA genotype appeared to be connected to higher values of glycemia, total cholesterol and LDL cholesterol.

## Introduction

Diabetes mellitus (DM) is a multifactorial disease characterized by chronic hyperglycemia and represents an important public health demand because it causes significant impacts on the quality of life and health management costs of the patients, especially when chronic complications occur. Microvascular complications are common and are related to several factors, especially diabetes duration and poor glycemic control.

Methylenetetrahydrofolate reductase (MTHFR) is an enzyme involved in the re-methylation of homocysteine (Hcy) in methionine cycle and catalyzes the reduction reaction of 5,10-methylenetetrahydrofolate to 5-methylenetetrahydrofolate. Thus, MTHFR function is one of the factors involved in the control of plasma levels of homocysteine. Elevated plasma levels of Hcy have been related to insulin resistance and to chronic complications such as diabetic retinopathy (DR) and diabetic nephropathy (DN) [1–3]. MTHFR is involved in the synthesis of the primary universal donor of methyl groups, *S*-adenosylmethionine (SAM), which is formed from methionine [4]. SAM is a substrate for the DNA methylation process that consists of an epigenetic mechanism that regulates the transcription of several genes and generally inhibits gene expression.

A previous study showed the association between the methylation profile in the *MTHFR* gene with the occurrence of chronic complications in diabetic patients. Briefly, comparison of the methylation profile of the MTHFR gene was performed in individuals with type 2 diabetes (DM2) who have been diagnosed with DM for 5–10 years. While the unmethylated profile was not identified in the analyzed samples, the partially methylated pattern predominated (~ 60%). The hypermethylated profile was associated with diabetic retinopathy (DR), but not with diabetic nephropathy (DN). Higher levels of total cholesterol and LDL cholesterol were identified in the hypermethylated profile only in DR patients samples [5].

Similarly, other reports, although controversial, describe gene polymorphisms that seem to interfere with the enzymatic activity of MTHFR and predispose individuals to diabetic complications. Studies indicate that the C677T polymorphism in the MTHFR gene, which is associated or not with inadequate glycemic control, may be linked to the progression of diabetic retinopathy [6, 7]. In addition, studies point to a significant association between this genotype and the development of nephropathy in diabetic patients [8, 9]. The A1298C polymorphism (rs1801131) has also been linked to the development of DN or macroalbuminuria, either alone or in combination with other alleles of interest, including C677T [10, 11]. However, the parallel effect of methylation profile and *MTHFR* polymorphisms on metabolic aspects in diabetic patients has never been analyzed.

Based on these facts, the objective of this work is to investigate in an unprecedented way the simultaneous relationship between *MTHFR* methylation profile and the C677T and A1298C polymorphisms and metabolic, inflammatory and oxidative stress factors related to microvascular complications in patients with diabetes for 5 to 10 years.

## Methodology

### Recruitment of subjects

Patients with type 2 diabetes mellitus DM2 of both sexes, older than 40 years, with at least 5 and at most 10 years of diagnostic, were recruited at the endocrinology, ophthalmology and nephrology services of the Lauro Wanderley University Hospital of the Federal University of Paraíba (HULW/UFPB) from August 2013 to November 2016. The subjects were divided into two groups: control group—patients without complications and group with complications—patients with retinopathy (DR) and/or nephropathy (DN).

### Ethical aspects

This project was approved by the Ethics Committee for Human Research of Federal University of Paraíba (Opinion No. 257.325; Report date: April 23, 2013). In addition, all procedures followed were in accordance with the institution’s ethical standards, conducted in compliance with Resolution 466/2012 of the National Health Council and the International Declaration of Helsinki.

### Clinical categorization of patients

The funduscopy examination was used to identify DR and 24-h urine albumin determination for identification of DN, the patients were included in the following clinical groups: 47 patients with complications (13 patients had RD, 25 had ND and 9 had both RD and ND) and 60 patients without complications (control), for a total of 107 patients.

The diagnosis of DR was based on ophthalmoscopy after pupil dilation with tropicamide 0.5%. Images of the retina (macula and central disc) were captured at a 45° angle with a fundus camera. All analyzes included in this study were performed by the same ophthalmologist. The photographs were analyzed according to the standards and recommendations of the Action to Control Cardiovascular Risk in Diabetes (ACCORD) and Early Treatment Diabetic Retinopathy Study (ETDRS). The presence of renal impairment was assessed by quantifying albumin in a 24-h urine sample. Microalbuminuria was defined as a urinary albumin concentration > 30 mg/L/24 h.

Clinical variables (age, date of diabetes diagnostic, glycemic control treatment, presence of hypertension, presence of dyslipidemia) were collected using an appropriate form.

### Collection of biological samples

For determination of albuminuria, patients received an appropriate container and were instructed to collect all urine for 24 h. They should then take the container to the researchers, ending the 24 h with the last collection in the hospital, at the time of the start of the exam the day before.

The blood was collected by venipuncture and samples were placed in different containers. For biochemical analysis in general, in the presence of clot activator, for determination of HbA1C in the presence of anticoagulant and for determination of glucose in the presence of anticoagulant sodium fluoride. The samples were centrifuged at a speed of 3000 rpm for 10 min at room temperature for separation of serum or plasma and subjected to analysis within 2 h after collection, except the sample for HbA_1_C that was analyzed in hemolyzed whole blood.

For DNA extraction, blood collection was performed by venous puncture in sterile tubes containing 7.2 mg of K_3_ EDTA. Blood samples were stored for up to 20 days at − 20 °C until DNA extraction was performed.

### Biochemical determinations

Determinations of fasting glucose (GLIC), serum creatinine (CREA-S), total cholesterol (TC), triglycerides (TRIG), HbA_1_C, C-reactive protein (CRP), alfa 1 acid glycoprotein (AGP), and high density lipoprotein cholesterol (HDL) were performed with commercial kits (Labtest^®^, Lagoa Santa, MG, Brazil) in automatic analyzer.

Light density lipoprotein cholesterol (LDL) concentration was determined using the Friedewald formula, where [LDL] = TC− [HDL] − [TRIG/5].

For determination of malondialdehyde (MDA), the method based on the reaction of thiobarbituric acid with hydroperoxides decomposition products was used. The total antioxidant capacity (TAC) of the serum was evaluated by the reduction of the 2,2-diphenyl-1-picryl-hydrazyl radical, which was measured by a colorimetric method in a spectrophotometer.

Urine was used to detect urinary albumin (M.ALB) using a commercial kit according to the guidelines recommended by the manufacturer (Labtest^®^, Lagoa Santa, MG, Brazil) in an automated analyzer. For the calculation of albumin excretion in 24 h, the value of the determination of albumin in the urine collected for 24 h (mg/dL) was multiplied by the total volume of urine collected in liters.

### DNA extraction for molecular analyzes

Leukocyte DNA was isolated using an protocol adapted from Miller et al. [5, 12].

### Determination of MTHFR genotypes C677T and A1298C

The presence of polymorphisms was determined using the restriction fragment length polymorphism (RFLP) technique by amplifying a fragment of the *MTHFR* gene by PCR using primers and temperature cycles described elsewhere [13, 14]. The 198 and 256 base pair fragments generated respectively by the amplification reaction of the polymorphisms C677T and A1298C were digested for 3 h with the endonucleases *Hinf*I (C677) and *Mob*II (A1298C) (Biolabs^®^) according to manufacturer’s guidelines. The RFLP profiles were generated by separation of DNA fragments in 15% polyacrylamide gel electrophoresis and observed by staining with silver nitrate or using the Gelred (Biotium^®^) intercalating dye followed by excitation by ultraviolet light in transilluminator. The genotypes 677 CC/CT/TT and 1298 AA/AC/CC were identified by the pattern of bands in the polyacrylamide gel according to the expected sizes described in the literature [13, 14].

### Analysis of the methylation profile in the *MTHFR* gene

Methylation analysis in the promoter of the *MTHFR* gene was performed using the methylation specific PCR (MSP) technique as previously described [5]. In short, the extracted leukocyte DNA was converted (500 ng) by sodium bisulfite protocol using EZ DNA Methylation ™ Kit (ZymoResearch) according to the manufacturer’s instructions. Methylation-specific PCR reactions were performed using 100 ng of bisulfite-transformed DNA, and specific pairs of primers for methylated and unmethylated targets in two separate amplification reactions. Methylated and unmethylated DNA (Cells-to-CpG ™ Methylated & Unmethylated DNA Control Kit, Life Technologies), which were modified as previously mentioned, and amplified by PCR, were analyzed together with the samples as a control for methylated and non-methylated conditions. Amplified PCR samples were loaded on 3% agarose gels with Gelred (Biotium^®^) and subjected to electrophoresis. The DNA bands were visualized with ultraviolet light. The samples were categorized as methylated (positive only for the methylated condition) or partially methylated (positive for methylated and non-methylated conditions). Non-methylated samples (positive only for the non-methylated condition) were not found in the population analyzed.

### Statistical analysis

The data were compiled in an Excel^®^ spreadsheet. Frequency was used for categorical variables and descriptive statistics for continuous variables. The Student’s t-test and Chi square test and, when necessary, the Mann–Whitney test and Fisher exact test were used in the program GraphPad, Instat, version 3.0. A post hoc test with total cholesterol results in the methylated profile was performed using the G* Power program 3.1.9.2. For all tests, p < 0.05 was used as the significance level.

**Table 1:** Demographic and clinical comparisons among the groups studied

	Control (n = 60)	With complications (n = 47)	*p*
Sex (M%)	15 (25%)	20 (42%)	0.054
Age (years)	56.9 ± 10.0	59.5 ± 8.1	0.1712
DM duration (years)	6.6 ± 2.1	7.6 ± 2.4	0.0266**
Oral hypoglycemic only	49 (81%)	27 (57%)	0.006*
Oral hypoglycemic + insulin/insulin only	7 (11.5%)	16 (34%)	0.0002*

Source: research data, 2018. *X ^2^ test; ** Mann–Whitney test

## Results

A total of 107 diabetic patients, all with diabetes diagnosed within the previous 5 to 10 years, were included in the following two experimental groups: 47 patients with complications (DR and/or DN) and 60 patients without complications (control). Comparison of the clinical and demographic data of the control groups and patients with complications (Table 1) showed that there are differences in diagnosis time that is slightly higher in the group of patients with complications (p = 0.026). The main difference between the groups is in the pharmacological treatment of glycemic control. While in the control group the use of oral hypoglycemic agents predominates (p = 0.006), in the group of patients with complications, the use of insulin associated with oral hypoglycemic agents is significantly higher (p = 0.0002).

Initially, there was an association between the genotypes and the clinical condition after evaluating the simultaneous effect of methylation profile and polymorphism in the *MTHFR* gene in all studied patients, independent of the clinical condition. For this analysis, the patients were divided into two categories according to the methylation profile of the *MTHFR* promoter: methylated and partially methylated. From the 107 samples analyzed, none presented the unmethylated profile of the MTHFR gene promoter, so the unmethylated category was not included in this study. The relationship of polymorphisms together with the methylation profile and the clinical conditions of the patients were analyzed, taking into account the following four groups: methylated with complications, methylated without complications, partially methylated with complications and partially methylated without complications.

### Influence of the methylation profile of *MTHFR* + polymorphism A1298C

Tables 2 and 3 describe relationships for the A1298C polymorphism. In Table 2, when all individuals were analyzed together, an association between the AA genotype and a hypermethylated promoter with higher glycemic values was identified (p = 0.03). A relationship between this same molecular profile and lipid profile was also observed, showing higher levels of TC (p = 0.0001) and LDL (p = 0.0006). A post hoc test with TC (methylated) was performed. At alpha significance level of 0.05, effect size and power (1-β err prob) were, respectively, 1.44 and 0.998. When the control and complication groups were analyzed separately (Table 3), it was observed that the effect of the genotype + hypermethylated profile appeared for glycemic control parameters fasting glycemia (p = 0.04) and HbA_1_C (p = 0.025) only in the control group. For the lipid profile parameters, while the relationship appeared in both groups for TC (p = 0.0049 and p = 0.0056, respectively), it remained only in the group with complications for LDL cholesterol (p = 0.002).

**Table 2:** Analysis of the association between the *MTHF* methylation profile and A1298C polymorphism of MTHFR and the biochemical, inflammatory and oxidative stress variables

		Methylated (42)			Partially methylated (65)		
		AA (22)	AC (17) + CC (3)	*p*	AA (36)	AC (23) + CC (6)	*p*
HbA1c	Mean ± SD Median	8.6 ± 1.7 8.4	7.9 ± 2.3 7.2	0.0718	7.9 ± 1.8 7.6	8.7 ± 1.8 9.0	0.0516
	Min.–Max.	5.7–13.0	5.3–14.4		4.1–12.7	4.3–11.2	
GLIC	Mean ± SD Median	186.1 ± 52.5 163.5	157.4 ± 51.5 135.0	0.0366*	159.8 ± 60.7 151.0	166.4 ± 70.0 145.0	0.8794
	Min.–Max.	121.0–301.0	85.0–282.0		72.0–308.0	85.0 ± 359.0	
TC	Mean ± SD Median	222.1 ± 47.6 214.3	164.6 ± 28.3 163.0	0.0001*	195.5 ± 56.5 187.0	195.7 ± 47.1 192.0	0.8225
	Min.–Max.	133.0–345.0	93.0–224.0		96.0 ± 320.0	127.0–316.0	
HDL	Mean ± SD Median	43.6 ± 9.4 42.0	46.1 ± 9.5 45.0	0.3918	46.1 ± 10.8 45.0	39.8 ± 11.6 39.0	0.0179*
	Min.–Max.	27.0–62.0	30.0–61.0		30.0–75.0	21.0–75.0	
LDL	Mean ± SD Median	134.8 ± 48.0 131.7	86.1 ± 30.7 84.7	0.0006*	119.0 ± 51.2 114.5	112.6 ± 50.6 110.4	0.7565
	Min.–Max.	29.0–227.0	29.4–158.4		46.8 ± 218.8	30.0–251.6	
TRIG	Mean ± SD Median	216.0 ± 129.1 196.5	184.0 ± 86.4 165.5	0.4350	177.8 ± 91.4 158.0	211.2 ± 106.8 177.0	0.1937
	Min.–Max.	56.0–650.0	55.0–398.0		67.0–488.0	53.0–484.0	
CREA-S	Mean ± SD Median	0.8 ± 0.3 0.8	0.8 ± 0.3 0.8	0.7529	0.9 ± 0.4 0.8	0.9 ± 0.3 0.8	0.4362
	Min.–Max.	0.4–1.4	0.4–1.7		0.5–2.2	0.5–2.2	
M. ALB	Mean ± SD Median	61.7 ± 140.5 18.0	20.4 ± 22.9 9.3	0.4651	79.8 ± 161.6 21.3	48.9 ± 129.9 7.2	0.0705
	Min.–Max.	1.0–650.0	1.0–76.0		1.0–650.0	1.0–525.0	
RCP	Mean ± SD Median	4.2 ± 3.7 3.8	3.3 ± 2.5 2.5	0.5839	3.6 ± 3.6 1.8	3.1 ± 2.9 2.2	0.7766
	Min.–Max.	0.4–13.3	0.4–9.5		0.3 ± 11.7	0.1–11.7	
AGP	Mean ± SD Median	95.0 ± 40.8 86.0	84.0–21.8 83.0	0.4652	74.5 ± 29.2 71.0	80.0 ± 25.8 76.0	0.3454
	Min.–Max.	59.0–263.0	55.0–140.0		4.0–176.0	21.0–172.0	
TAC	Mean ± SD Median	40.8 ± 28.0 42.0	55.0 ± 27.0 61.0	0.1337	24.8 ± 25.6 12.0	26.9 ± 25.0 13.0	0.4800
	Min.–Max.	5.0–91.0	8.0–94.0		2.0–96.0	4.0–84.0	
MDA	Mean ± SD Median	3.4 ± 1.1 3.7	3.9 ± 0.6 3.7	0.3579	3.5 ± 1.3 3.7	3.3 ± 1.4 3.4	0.4843
	Min.–Max.	1.1–4.9	3.1–5.1		1.0–6.2	1.4–6.3	

*HbA1C* (%) glycated haemoglobin, *GLIC* (mg/dL) fasting glycemia, *TC* (mg/dL) total cholesterol, *HDL* (mg/dL) high density lipoprotein, *LDL* (mg/dL) light density lipoprotein cholesterol, *TRIG* (mg/dL) triglycerides, *CREA*-*S* (mg/dL) serum creatinine, *M. ALB* (mg/dL) 24 h albumin excreted in the urine, *RCP* (mg/dL) reactive C protein, *AGP* (mg/dL) alfa 1 acid glycoprotein, *TAC* (%) total antioxidant capacity, *MDA* (µM) malondialdehyde

* Statistically significant (p < 0.05), Mann–Whitney test

**Table 3:** Analysis of the relationship between the MTHFR methylation pattern and the A1298C polymorphism and biochemical, inflammatory and oxidative stress variables

		With complications (20)			Control (22)			With complications (27)			Control (38)		
		Methylated AA (13)	Methylated AC (5) + CC (2)	*p*	Methylated AA (9)	Methylated AC (12) + CC (1)	*p*	Partially Methylated AA (17)	Partially Methylated AC (9) + CC (1)	*p*	Partially _Methylated AA_ (19)	Partially Methylated AC (14) + CC (15)	*p*
HbA1c	Mean ± SD Median	8.5 ± 1.9 8.1	9.4 ± 3.2 7.2	> 0.9999	8.6 ± 1.3 8.6	7.2 ± 1.1 7.2	0.0253*	8.3 ± 1.7 8.0	9.0 ± 1.5 9.0	0.2094	7.6 ± 1.9 7.5	8.6 ± 1.9 9.2	0.0932
	Min.–Max.	5.7‒13.00	6.9‒14.4		6.7‒11.1	5.3‒9.4		6.1‒12.0	7.1‒11.0		4.1‒12.7	4.3‒11.2	
GLIC	Mean ± SD Median	182.2 ± 54.0 160.0	169.0 ± 47.5 172.0	0.7573	191.8 ± 53.0 200.0	151.1 ± 54.3 132.0	0.0489*	153.7 ± 65.2 136.0	163.5 ± 76.1 135.0	0.7065	165.3 ± 57.5 162.0	168.0 ± 68.8 151.0	0.8040
	Min.–Max.	123.0‒301.0	117.0‒248.0		121.0‒270.0	85.0‒282.0		80.0‒308.0	97.0‒359.0		72.0‒303.0	85.0 ± 348.0	
TC	Mean ± SD Median	230.1 ± 51.0 214.0	168.7 ± 27.6 164	0.0049*	210.7 ± 42.5 200.0	162.3 ± 29.4 162.0	0.0056*	206.5 ± 61.7 187.0	208.0 ± 62.7 209.5	0.9001	185.6 ± 50.9 187.0	189.2 ± 36.9 185.0	0.8040
	Min.–Max.	159‒345	132‒211		133.0‒270.0	93.0‒224.0		139.0‒320.0	129.0‒316.0		96.0‒283.0	127.0‒257.0	
HDL	Mean ± SD Median	40.3 ± 8.1 39.0	47.3 ± 8.2 47.0	0.1043	48.2 ± 9.7 49.0	45.5 ± 10.4 42.0	0.5258	43.6 ± 12.4 40.0	40.0 ± 12.6 42.0	0.4217	48.4 ± 9.0 58.0	39.7 ± 11.5 39.0	0.0044*
	Min.–Max.	27.0‒56.0	33.0‒57.0		32.0‒62.0	30.0‒61.0		30.0‒75.0	21.0‒54.0		33.0‒61.0	23.0‒75.0	
LDL	Mean ± SD Median	142.3 ± 54.0 140.4	77.8 ± 18.2 68.4	0.0024*	123.8 ± 38.1 123.0	90.6 ± 35.6 92.0	0.0825	129.8 ± 53.9 118.0	118.8 ± 69.0 116.7	0.2685	109.3 ± 48.1 101.0	109.4 ± 39.6 110.4	0.8153
	Min.–Max.	29.0‒227.0	62.0‒112.6		63.4‒184.0	29.4‒158.4		61.8‒218.8	42.0‒251.6		46.8‒209.9	30.0‒181.0	
TRIG	Mean ± SD Median	231.5 ± 157.0 200.0	218.3 ± 114.5 172.0	0.8773	193.4 ± 76.3 193.0	165.5 ± 65.0 158.0	0.4310	188.4 ± 77.5 165.0	230.8 ± 108.0 201.5	0.1319	168.4 ± 103.5 146.0	200.8 ± 107.7 168.0	0.2801
	Min.–Max.	77.0‒650.0	55.0‒398.0		56.0‒290.0	80.0‒292.0		80.0‒356.0	67.0‒464.0		67.0‒488.0	53.0 ± 484.0	
CREA-S	Mean ± SD Median	0.9 ± 0.3 0.9	0.9 ± 0.3 0.8	0.7573	0.7 ± 0.2 0.7	0.8 ± 0.3 0.7	0.9479	1.0 ± 0.3 1.0	1.1 ± 0.5 1.1	0.8018	0.9 ± 0.4 0.7	0.7 ± 0.1 0.7	0.8955
	Min.–Max.	0.4‒1.4	0.5 ± 1.3		0.6‒1.2	0.4‒1.8		0.5‒1.8	0.6‒2.2		0.4‒2.2	0.5‒1.0	
M. ALB	Mean ± SD Median	99.9 ± 175.1 40.0	41.3 ± 27.2 46.0	0.8773	6.7 ± 6.8 3.0	9.2 ± 8.4 6.0	0.4620	156.8 ± 212.3 46.0	128.2 ± 204.2 33.6	0.3033	10.8 ± 9.2 10.0	7.2 ± 7.9 4.0	0.2992
	Min.–Max.	1.0‒650.0	3.0 ± 76.0		1.0‒20.0	1.0‒26.0		7.0‒650.0	1.0‒525.0		1.0‒25.0	1.0‒28.0	
CRP	Mean ± SD Median	4.8 ± 3.3 4.9	3.6 ± 2.9 2.1	0.5358	3.4 ± 4.1 2.3	3.1 ± 2.4 2.5	0.6948	3.7 ± 3.8 1.6	2.6 ± 1.8 2.1	0.9411	3.6 ± 3.6 1.9	3.4 ± 3.4 3.3	0.7481
	Min.–Max.	0.6‒11.9	1.0‒8.2		0.4‒13.3	0.4‒9.5		0.4‒11.5	0.7‒6.2		0.3‒11.7	0.1‒11.7	
AGP	Mean ± SD Median	101.0 ± 51.9 85.0	81.1 ± 21.5 72.0	0.4219	87.0 ± 17.8 87.0	85.6 ± 22.6 84.0	0.7438	72.9 ± 36.1 69.0	78.6 ± 38.1 72.5	0.4820	76.0 ± 22.3 72.0	80.8 ± 16.7 77.0	0.6934
	Min.–Max.	72.0‒263.0	57.0‒109.0		59.0‒118.0	55.0‒140.0		16.0‒176.0	21.0‒172.0		4.0‒105.0	52.0‒121.0	
TAC	Mean ± SD Median	37.0 ± 24.9 37.0	51.3 ± 30.3 63.0	0.3104	45.8 ± 32.4 42.0	57.0 ± 26.1 59.0	0.4425	15.8 ± 12.4 12.0	29.4 ± 26.5 18.0	0.1079	32.9 ± 31.5 19.0	25.6 ± 24.8 12.0	0.7041
	Min.–Max.	9.0‒72.0	9.0‒87.0		5.0‒91.0	8.0‒94.0		2.0‒46.0	8.0‒80.0		6.0‒96.0	4.0‒84.0	
MDA	Mean ± SD Median	3.0 ± 1.2 3.4	4.0 ± 0.7 4.1	0.0811	4.1 ± 0.7 4.0	3.9 ± 0.7 3.6	0.3851	3.7 ± 1.3 3.7	3.2 ± 1.7 2.9	0.4821	3.4 ± 1.2 3.8	3.4 ± 1.2 3.4	0.8724
	Min.–Max.	1.1‒4.8	3.1‒4.8		2.8‒4.9	3.1‒5.1		1.0‒6.2	1.4‒6.3		1.4‒5.3	1.4‒5.6	

*HbA1C* (%) glycated haemoglobin, *GLIC* (mg/dL) fasting glycemia, *TC* (mg/dL) total cholesterol, *HDL* (mg/dL) high density lipoprotein, *LDL* (mg/dL) light density lipoprotein cholesterol, *TRIG* (mg/dL) triglycerides, *CREA*-*S* (mg/dL) serum creatinine, *M. ALB* (mg/dL) 24 h albumin excreted in the urine, *RCP* (mg/dL) reactive C protein, *AGP* (mg/dL) alfa 1 acid glycoprotein, *TAC* (%) total antioxidant capacity, *MDA* (µM) malondialdehyde

* Statistically significant (p < 0.05), Mann–Whitney test

### Influence of the methylation profile of *MTHFR* + C677T polymorphism

For the C677T polymorphism, the genotypic distribution was fairly balanced between the with complications and without complications phenotypic groups (data not show). For Table 4, analyzing all individuals (complicated + uncomplicated) there were no significant results. In Table 5, analyzing the methylation profile and clinical genotype, only the intersection between CC and TC + TT in the hypermethylated group for creatinine was significant (p = 0.0040). This trend continued when the division of the methylation profile was funneled between the with complications and control groups (p = 0.0020).

**Table 4:** Analysis of the relationship between the *MTHFR* methylation pattern and the C677T polymorphism of MTHFR and biochemical, inflammatory and oxidative stress variables

		Methylated (42)			Partially methylated (65)		
		CC (21)	TC (18) + TT (3)	*p*	CC (30)	TC (33) + TT (2)	*p*
GLIC	Mean ± SD Median	164.8 ± 56.3 139.0	180.1 ± 50.5 167.0	0.2273	158.2 ± 59.3 147.0	166.7 ± 69.4 152.0	0.6499
	Min.–Max.	85.0–301.0	121.0–282.0		85.0–303.0	72.0–359.0	
HbA1c	Mean ± SD Median	8.5 ± 2.6 7.9	8.0 ± 1.2 8.0	0.9599	8.3 ± 1.7 8.3	8.3 ± 2.0 8.0	0.8332
	Min.–Max.	5.3–14.4	5.7–11.1		4.1–110	4.7–12.7	
TC	Mean ± SD Median	185.8 ± 39.3 93.0	203.7 ± 56.2 133.0	0.5629	204.1 ± 56.8 187.0	188.2 ± 47.4 187.0	0.3570
	Min.–Max.	93.0–272.0	133.0–145.0		127.0–320.0	96.0–316.0	
HDL	Mean ± SD Median	45.0 ± 9.6 46.0	44.6 ± 9.4 43.0	0.8800	42.1 ± 12.0 41.5	44.3 ± 11.2 43.0	0.3569
	Min.–Max.	30.0–61.0	27.0–62.0		23.0–75.0	21.0–75.0	
LDL	Mean ± SD Median	109.3 ± 37.4 112.6	113.9 ± 56.1 103.6	0.9398	127.8 ± 52.2 117.5	106.2 ± 47.8 101.8	0.1388
	Min.–Max.	29.4–177.0	29.0–227.0		46.8–251.6	30.0–215.6	
TRIG	Mean ± SD Median	172.2 ± 78.6 165.0	229.2 ± 131.4 207.0	0.1189	179.7 ± 87.5 170.5	203.8 ± 108.2 181.0	0.4454
	Min.–Max.	55.0–329.0	56.0–650.0		67.0–488.0	53.0–484.0	
CREA-S	Mean ± SD Median	1.0 ± 0.3	0.7 ± 0.2	0.0080*	0.9 ± 0.4 0.8	0.9 ± 0.4 0.8	0.7372
	Min.–Max.	0.5–1.8	0.4–1.2		0.5–2.2	0.5–2.2	
M. ALB	Mean ± SD Median	35.5 ± 50.4 15.0	48.7 ± 139.6 13.0	0.5627	66.4 ± 146.2 11.0	65.7 ± 151.7 18.0	0.8025
	Min.–Max.	1.0–205.0	1.0–650.0		1.0–525.0	1.0–650.0	
CRP	Mean ± SD Median	3.6 ± 3.1 2.5	3.9 ± 3.3 4.1	0.8144	3.9 ± 3.6 2.8	3.0 ± 3.0 1.8	0.2496
	Min.–Max.	0.6–11.9	0.4–13.3		0.3–11.7	0.1–11.7	
AGP	Mean ± SD Median	96.0 ± 44.3 89.5	83.7 ± 15.3 84.0	0.4652	80.9 ± 22.6 75.0	73.6 ± 31.3 70.0	0.2089
	Min.–Max.	55.0–263.0	56.0–118.0		52.0–172.0	4.0–176.0	
TAC	Mean ± SD Median	54.2 ± 25.1 57.0	41.5 ± 29.9 42.0	0.2458	27.6 ± 27.8 13.0	24.2 ± 22.9 12.0	0.6262
	Min.–Max.	8.0–94.0	5.0–91.0		4.0–96.0	2.0–82.0	
MDA	Mean ± SD Median	3.6 ± 1.1 3.7	3.7 ± 0.8 3.7	0.7916	3.5 ± 1.3 3.4	3.4 ± 1.3 3.7	0.8642
	Min.–Max.	1.1–5.1	2.3–4.9		1.4–6.3	1.0–6.2	

*HbA1C* (%) glycated haemoglobin, *GLIC* (mg/dL) fasting glycemia, *TC* (mg/dL) total cholesterol, *HDL* (mg/dL) high density lipoprotein, *LDL* (mg/dL) light density lipoprotein cholesterol, *TRIG* (mg/dL) triglycerides, *CREA*-*S* (mg/dL) serum creatinine, *M. ALB* (mg/dL) 24 h albumin excreted in the urine, *RCP* (mg/dL) reactive C protein, *AGP* (mg/dL) alfa 1 acid glycoprotein, *TAC* (%) total antioxidant capacity, *MDA* (µM) malondialdehyde

* Statistically significant (p < 0.05), Mann–Whitney test

**Table 5:** Analysis of the relationship between the *MTHFR* methylation pattern and the C677C polymorphism of MTHFR and biochemical, inflammatory and oxidative stress variables associated with clinical condition

		With complications (20)			Control (22)			With complications (27)			Control (38)		
		Methylated CC (11)	MethylatedTC (6) + TT (3)	*p*	Methylated CC (10)	Methylated TC (12)	*p*	Partially Methylated CC (10)	Partially MethylatedTC (16) + TT (1)	*p*	Partially Methylated CC (20)	Partially MethylatedTC (17) + TT (1)	*p*
HbA1c	Mean ± SD Median	9.7 ± 2.9 9.0	7.8 ± 1.1 7.7	0.3231	7.2 ± 1.3 7.2	8.1 ± 1.3 8.0	0.1984	8.4 ± 1.4 8.2	8.6 ± 1.8 8.0	0.9399	8.2 ± 1.9 8.3	8.0 ± 2.1 7.6	0.5785
	Min.–Max.	6.4–14.4	5.7–9.6		5.3‒9.3	6.5–11.1		6.8–11.0	6.1–12.0		4.1–10.5	4.7–12.7	
GLIC	Mean ± SD Median	183.0 ± 60.6 160.0	171.0 ± 38.7 167.0	0.9408	144.7 ± 46.1 131.5	186.9 ± 58.6 172.0	0.0750	139.6 ± 48.3 126.5	167.8 ± 76.9 150.0	0.4074	167.5 ± 63.1 171.0	165.7 ± 63.7 151.0	0.7039
	Min.–Max.	117.0–301.0	123.0–243.0		85.0–226.0	12.01‒282.0		96.0–262.0	80.0–359.0		85.0–303.0	72.0–348.0	
TC	Mean ± SD Median	194.3 ± 40.3 202.0	226.0 ± 62.9 204.0	0.3422	176.3 ± 37.9 174.0	186.9 ± 46.4 169.0	0.9999	220.8 ± 72.0 206.5	199.0 ± 54.1 187.0	0.5807	195.8 ± 47.4 185.5	178.1 ± 38.8 188.5	0.3495
	Min.–Max.	132.0–273.0	159.0–345.0		93.0‒226.0	133.0‒270.0		129.0–320.0	131.0–316.0		127.0–283.0	96.0–238.0	
HDL	Mean ± SD Median	44.9 ± 9.8 47.0	40.2 ± 6.4 41.0	0.3050	45.1 ± 9.9 44.0	47.9 ± 10.2 48.0	0.6744	45.9 ± 15.5 49.0	40.1 ± 10.0 39.0	0.4820	40.2 ± 9.7 40.0	48.3 ± 11.1 46.5	0.0273*
	Min.–Max.	30.0–57.0	27.0–50.0		30.0‒61.0	32.0‒62.0		29.0–75.0	21.0–57.0		23.0–60.0	30.0 ± 75.0	
LDL	Mean ± SD Median	111.7 ± 37.5 112.6	129.6–71.0 103.6	0.9999	106.6 ± 38.9 109.3	102.1 ± 41.4 92.7	0.5824	143.5 ± 63.1 127.4	115.3 ± 5.4 111.0	0.3338	120.0 ± 45.5 116.1	97.5 ± 38.9 101.5	0.1933
	Min.–Max.	62.0–177.0	29.0–227.0		29.4‒158.4	52.8—184		65.6–251.6	42.0–215.6		46.8–209.9	30.0–181.0	
TRIG	Mean ± SD Median	189.0 ± 93.1 170.0	273.2 ± 177.9 207.0	0.2947	153.7 ± 58.0 146.0	196.2 ± 74.7 201.5	0.1593	157.0 ± 54.7 174.5	231.8 ± 96.9 251.0	0.0459*	191.1 ± 99.3 166.5	177.4 ± 114.3 148.4	0.4385
	Min.–Max.	55.0–329.0	82.0–650.0		80.0‒272.0	56.0‒292.0		67.0–243.0	80.0–464.0		67.0–488.0	53.0–484.0	
CREA-S	Mean ± SD Median	1.0 ± 0.3 1.0	0.8 ± 0.2 0.9	0.2947	0.9 ± 0.3 0.8	0.6 ± 0.2 0.6	0.0020*	1.2 ± 0.4 1.0	1.0 ± 0.4 1.0	0.5139	0.8 ± 0.3 0.7	0.8 ± 0.4 0.7	0.6089
	Min.–Max.	0.5–1.4	0.6–1.1		0.7‒1.7	0.4‒1.2		0.7–2.2	0.5–1.8		0.5–1.8	0.5–2.2	
M. ALB	Mean ± SD Median	60.2 ± 60.0 43.0	102.8 ± 207.0 25.0	0.8238	8.2 ± 7.5 7.2	8.1 ± 8.2 4.6	0.9737	180.4 ± 216.7 52.0	126.0 ± 203.1 42.5	0.5701	9.3 ± 8.8 6.6	8.6 ± 8.7 4.0	0.3719
	Min.–Max.	3.0–205.0	1.0–650.0		1.0‒24.0	1.0‒26.0		1.0–525.0	4.1–650.0		1.0–28.0	1.0–22.0	
CRP	Mean ± SD Median	3.8 ± 3.7 2.6	5.0 ± 2.5 6.4	0.2110	3.3 ± 2.5 2.5	3.1 ± 3.7 2.0	0.5387	3.6 ± 3.3 2.2	3.0 ± 3.2 1.8	0.3595	4.0 ± 3.8 3.6	2.9 ± 3.0 2.1	0.3571
	Min.–Max.	0.6–11.9	1.2–7.7		0.6–9.5	0.4–13.3		0.9–11.5	0.4–9.6		0.3–11.7	0.1–11.6	
AGP	Mean ± SD Median	101.9 ± 59.3 89.5	84.6 ± 11.7 84.0	0.7131	90.0 ± 23.2 89.5	83.0 ± 18.0 82.5	0.5387	82.3 ± 32.5 75.0	70.7 ± 38.5 68.0	0.2186	80.2 ± 16.7 74.5	76.3 ± 23.5 77.5	0.6504
	Min.–Max.	57.0–263.0	68.0–102.0		55.0–140.0	56.0–118.0		60.0–172.0	16.0–176.0		52.0–121.0	4.0–111.0	
TAC	Mean ± SD Median	51.0 ± 19.0 52.5	32.6 ± 32.4 13.0	0.1564	57.5 ± 30.7 64.5	48.2 ± 27.5 47.5	0.5387	31.4 ± 26.1 22.0	14.6 ± 11.2 11.0	0.0195*	25.7 ± 29.1 12.0	33.2 ± 27.4 15.5	0.2728
	Min.–Max.	15.0–75.0	9.0–87.0		8.0–94.0	5.0–91.0		8.0–80.0	2.0–44.0		4.0–96.0	6.0–82.0	
MDA	Mean ± SD Median	3.3 ± 1.4 3.8	3.5 ± 0.8 3.6	0.9013	3.9 ± 0.6 3.7	3.9 ± 0.7 4.0	0.9474	3.6 ± 1.4 3.3	3.4 ± 1.6 3.7	0.7632	3.4 ± 1.2 3.6	3.4 ± 1.1 3.6	0.9185
	Min.–Max.	1.1–4.8	2.3–4.8		3.2–5.1	2.8–4.9		1.7–6.3	1.0–6.2		1.4–5.6	1.5–5.3	

*HbA1C* (%) glycated haemoglobin, *GLIC* (mg/dL) fasting glycemia, *TC* (mg/dL) total cholesterol, *HDL* (mg/dL) high density lipoprotein, *LDL* (mg/dL) light density lipoprotein cholesterol, *TRIG* (mg/dL) triglycerides, *CREA*-*S* (mg/dL) serum creatinine, *M. ALB* (mg/dL) 24 h albumin excreted in the urine, *RCP* (mg/dL) reactive C protein, *AGP* (mg/dL) alfa 1 acid glycoprotein, *TAC* (%) total antioxidant capacity, *MDA* (µM) malondialdehyde

* Statistically significant (p < 0.05), Mann–Whitney test

In the group with complications, the triglyceride values were higher in the partially methylated group profile in the presence of CT + TT (0.04) genotypes, while the TAC was higher in the same profile but in the presence of the CC genotype (p = 0.01). In addition, the lipid profile was also affected, with the partially methylated group presenting higher levels of HDL (p = 0.0273) in the control group in the presence of CT + TT genotypes.

### Influence of the methylation profile of *MTHFR* + haplotype C677T/A1298C

Table 6 shows the results of intersections between the haplotypes C677T and A1298C, divided by the methylation profile (hypermethylated and partially methylated, respectively). For the hypermethylated group, glycemia was significant between 677CC/1298AA and 677CC/1298AC + CC (p = 0.0077), with values from the latter group (mean = 139.9 and median = 129.0) being significantly improved relative to the former (mean = 205.1 and median = 214.0). For total cholesterol (p = 0.0024) and LDL (p = 0.0060), the same trend was observed, with lower values for those with 677CC/1298AC + CC. In the relationship between the partially methylated individuals and the haplotype no significant difference was found.

**Table 6:** Analysis of the relationship between the *MTHFR* methylation pattern and the A1298C + C677T polymorphism of MTHFR and biochemical, inflammatory and oxidative stress variables

		Hypermethylated						Partially methylated					
		677CC/1298AA (8)	677CC/1298AC (10) + CC (3)	*p*	677CT (11) + TT (3)/1298AA (14)	677CT/1298AC (7)	*p*	677CC/1298AA (13)	677CC/298AC (12) + CC (5)	*P*	677CT (21) + TT (2)/1298AA (23)	677CT/1298AC (11)	*P*
HbA1c	Mean ± SD Median	9.4 ± 2.0 9.2	7.9 ± 2.8 7.1	0.0638	8.0 ± 1.3 8.1	7.9 ± 1.2 7.5	0.7653	7.8 ± 1.5 7.8	8.6 ± 1.8 9.2	0.1547	8.0 ± 2.0 7.5	8.9 ± 1.8 8.6	
	Min.–Max.	6.4‒3.0	5.3‒14.4		5.7‒1.1	6.5‒9.6		4.1‒10.3	4.3‒11.0		4.7‒12.7	5.7‒11.2	0.1262
GLIC	Mean ± SD Median	205.1 ± 54.6 214.0	139.9 ± 42.4 129.0	0.0077*	175.3 ± 50.0 152.0	189.7 ± 54.1 192.0	0.5506	166.8 ± 61.1 165.0	151.6 ± 58.9 141.0	0.3682	155.9 ± 61.4 152.0	187.4 ± 81.4 162.5	
	Min.–Max.	133.0‒301.0	85.0‒248.0		121.0‒270.0	123.0‒282.0		95.0‒303.0	85.0‒265.0		72.0‒308.0	123.0‒359.0	0.2892
COL T	Mean ± SD Median	217.0 ± 26.5 214.3	166.5 ± 33.4 163.0	0.0024*	225.1 ± 57.1 212.5	160.9 ± 16.4 157.0	0.0031*	204.4 ± 65.3 187.0	203.9 ± 51.4 186.0	0.9016	190.4 ± 51.7 186.0	184.0‒39.5 192.5	
	Min.–Max.	185.0‒273.0	93.0‒224.0		133.0‒345.0	143.0‒192.0		128.0‒320.0	127.0‒316.0		96.0‒316.0	131.0‒246.0	0.9446
HDL	Mean ± SD Median	44.3 ± 9.1 47.7	45.4 ± 10.2 44.0	0.9711	43.1 ± 9.9 41.0	47.6 ± 8.4 47.0	0.2629	46.4 ± 13.6 48.0	38.9 ± 9.8 39.0	0.1214	46.0 ± 9.2 45.0	41.2 ± 14.2 39.0	
	Min.–Max.	30.0‒56.0	30.0‒61.0		27.0‒62.0	37.0‒58.0		30.0‒75.0	23.0‒54.0		30.0‒61.0	21.0‒75.0	0.1396
LDL	Mean ± SD Median	135.9 ± 27.5 131.2	92.5 ± 33.5 92.6	0.0060*	134.1 ± 57.6 133.2	73.5 ± 21.5 65.8	0.0125*	125.9 ± 62.0 118.0	129.2 ± 45.2 117.0	0.6801	115.0 ± 45.1 111.0	89.2 ± 50.2 69.2	
	Min.–Max.	101.4‒177.0	29.4‒158.4		29.0‒227.0	52.8‒116.0		46.8‒218.0	65.6‒251.6		57.2‒215.6	30.0‒181.0	0.1307
TRIG	Mean ± SD Median	184.2 ± 89.5 167.0	164.8 ± 73.9 165.0	0.7172	234.1 ± 147.1 203.5	219.6 ± 102.3 216.0	0.9710	180.8 ± 112.3 146.0	178.9 ± 66.5 176.0	0.6303	176.1 ± 79.9 160.0	256.8 ± 136.9 213.5	
	Min.–Max.	77.0‒329.0	55.0‒327.0		56.0‒650.0	116.0‒398.0		67.0‒488.0	67.0‒297.0		72.0‒356.0	53.0‒484.0	0.1024
CREA-S	Mean ± SD Median	0.9 ± 0.3 0.8	0.9 ± 0.3 0.9	0.9718	0.8 ± 0.2 0.7	0.6 ± 0.1 0.6	0.0524	0.9 ± 0.4 0.8	0.9 ± 0.4 0.8	0.7695	0.9 ± 0.4 0.9	0.8 ± 0.2 0.7	
	Min.–Max.	0.6‒1.4	0.5‒1.7		0.4‒1.2	0.4‒0.8		0.5‒1.8	0.5‒2.2		0.5‒2.2	0.6‒1.3	0.5781
M. ALB	Mean ± SD Median	64.0 ± 70.8 41.5	17.9 ± 20.8 9.0	0.0647	60.5 ± 170.8 11.5	25.2 ± 27.4 16.2	0.5757	61.53 ± 119.8 24.0	70.0 ± 167.1 7.2	0.4638	90.1 ± 182.8 21.0	18.9 ± 25.6 5.8	
	Min.–Max.	1.0‒205.0	1.0‒67.0		1.0‒650.0	1.0‒76.0		1.0‒439.0	1.0‒525.0		1.0‒650.0	1.0 ± 84.7	0.1216
CRP	Mean ± SD Median	4.4 ± 3.7 3.8	3.1 ± 2.8 2.5	0.3929	4.1 ± 3.8 3.3	3.5 ± 2.2 4.2	0.8557	4.2 ± 4.1 1.9	3.7 ± 3.3 3.4	0.9016	3.3 ± 3.4 1.7	2.3 ± 2.2 1.9	
	Min.–Max.	0.6 ± 11.9	0.6 ± 9.5		0.4‒13.3	0.4‒6.9		0.3‒11.5	0.3‒11.7		0.3‒11.7	0.1‒8.0	0.5257
AGP	Mean ± SD Median	111.7 ± 67.4 95.0	87.4 ± 24.5 88.0	0.7573	86.6 ± 15.0 85.0	77.9 ± 15.3 73.0	0.2793	77.1 ± 12.5 72.0	83.8 ± 28.1 76.0	0.7063	73.0 ± 35.6 69.0	74.6 ± 22.3 74.0	
	Min.–Max.	72.0‒263.0	55.0‒140.0		59.0‒118.0	56.0‒102.0		60.0‒102.0	52.0‒172.0		4.0‒176.0	21.0‒111.0	0.5901
TAC	Mean ± SD Median	44.7 ± 20.2 51.0	59.4 ± 26.6 69.0	0.1223	38.8 ± 31.7 29.0	46.9 ± 27.7 51.0	0.6015	29.9 ± 28.4 22.0	25.9 ± 28.0 13.0	0.4636	21.9 ± 23.9 11.0	28.4 ± 20.9 17.5	
	Min.–Max.	8.0‒68.0	8.0‒94.0		9.0‒87.0	9.0‒87.0		6.0‒96.0	84.0‒13.0		2.0‒82.0	8.0‒60.0	0.1491
MDA	Mean ± SD Median	2.9 ± 1.4 3.7	4.0 ± 0.7 3.8	0.1922	3.7 ± 0.9 3.8	3.7 ± 0.5 3.6	0.7990	3.5 ± 1.1 3.9	3.4 ± 1.4 3.4	0.6603	3.5 ± 1.4 3.7	3.2 ± 1.3 3.4	
	Min.–Max.	1.1‒4.2	3.2‒5.1		2.3‒4.9	3.1‒4.3		1.4‒4.9	1.4‒6.3		1.0‒6.2	1.4‒5.3	0.5900

*HbA1C* (%) glycated haemoglobin, *GLIC* (mg/dL) fasting glycemia, *TC* (mg/dL) total cholesterol, *HDL* (mg/dL) high density lipoprotein, *LDL* (mg/dL) light density lipoprotein cholesterol, *TRIG* (mg/dL) triglycerides, *CREA*-*S* (mg/dL) serum creatinine, *M. ALB* (mg/dL) 24 h albumin excreted in the urine, *RCP* (mg/dL) reactive C protein, *AGP* (mg/dL) alpha 1 acid glycoprotein, *TAC* (%) total antioxidant capacity, *MDA* (µM) malondialdehyde

* Statistically significant (p < 0.05), Mann–Whitney test

## Discussion

The main result of this work is the simultaneous effect of the hypermethylation and A1298C polymorphism of the *MTHFR* gene on lipid parameters and glycemic control in diabetic patients.

The *MTHFR* gene is located on the short arm of chromosome 1 (1p26.3), has 11 exons and is expressed through the production of three transcripts of different sizes in the human species, suggesting the involvement of complex gene regulation mechanisms [15]. Analysis of the promoter region by computational analysis revealed the presence of two CpG islands with potential binding sites for various transcription factors, suggesting that transcriptional control of the production of this enzyme may undergo methylation control [16].

Few studies have analyzed the effects of the methylation profile of *MTHFR* and the occurrence of complications in diabetes. A recent study in which samples of healthy, diabetic, early-stage and advanced-stage DN patients were analyzed an association between *MTHFR* demethylation and DN morbidity was identified in diabetic patients. While the healthy control group did not have demethylated specimens, the diabetic group and the group with early DN showed a higher level of demethylated samples, and the clinical DN group did not present methylated samples [17]. In addition, these results showed an association between increasing levels of homocysteine (Hcy) and demethylation of *MTHFR*. This effect of the concentration of HCY on the methylation profile of *MTHFR* has already been demonstrated in in vitro experiments with human muscle cells, which revealed an even higher production of transcripts in the demethylated *MTHFR* pattern [18]. The authors argue that there may be a compensatory effect causing *MTHFR* demethylation when HCY is elevated to increase the expression of the enzyme and consequently the conversion of Hcy to methionine. This effect would be evident in the samples of patients with clinical DN, who had high levels of HCY and demethylated profiles [17]. Another study that analysed the relationship between *MTHFR* methylation and end-stage renal disease, not specifically in DN, has been reported an association between methylation and higher levels of total cholesterol and LDL cholesterol [19]. Diabetic retinopathy and higher levels of total cholesterol and LDL cholesterol has also been associated with the hypermethylated *MTHFR* pattern in patients with a diagnosis time of diabetes of 5 to 10 years [5], although the relationship has not been identified in samples from patients with DN.

In this work the objective was to simultaneously analyze the effect of the methylation profile and polymorphisms in the *MTHFR* gene on biochemical variables taking into consideration the clinical condition of the diabetic patient.

Two polymorphisms in MTHFR, C677T and A1298C, have been most studied because they affect enzymatic activity. The C677T polymorphism, which causes an alanine substitution by valine (Ala222Val), occurs in exon 4 of the *MTHFR* gene and results in enzyme thermolability and decreased activity. It has been shown that 677TT homozygotes and 677CT heterozygotes have approximately 70% and 35% reduced MTHFR activity, respectively [13, 20]. The 677TT genotype is associated with global hypomethylation in the healthy cell genome of cancer patients [21].

The A1298C polymorphism results in the substitution of glutamic acid for alanine (Glu429Ala), and although the homozygote showed a slight reduction in enzymatic activity, it had no effect on Hcy concentration [14]. This polymorphism is located in the regulatory domain of the enzyme responsible for binding to NADPH and S-adenosylmethionine [22].

In this study, while the C677T polymorphism did not appear to affect the distribution of the patients in the with complications and without complications groups, the 1298C allele genotypes (AC + CC) appeared in a higher percentage in the group without complications in diabetes, although without statistical significance, suggesting a protective effect of the C allele. This is the allele that appears to have a minor impact on MTHFR activity, although studies have shown that individuals with the 677CC/1298CC haplotype have lower homocysteine levels than do those with the 677CC/1298AA haplotype [23]. However, the allele 1298C has appeared as a protective factor for other medical conditions, such as congenital heart defects [24]. A possible explanation for this fact, noted by the authors of the cited articles, is the present linkage disequilibrium between the 677T allele, which causes significant reduction in the enzymatic activity and the allele in question, 1298C, which would result in a false protection effect of the mutant allele 1298C. The study further proposes that the 1298C allele may appear in linkage disequilibrium with another yet unrecognized polymorphism of MTHFR. In addition, the 1298C allele was cited as a protective factor for folate deficiency and related to higher levels of this nutrient in comparison with the 1298AA genotype [20, 25]. A possible explanation for these findings is related to the location of the polymorphism, which affects the binding site for the negative allosteric effector *S*-adenosylmethionine, which could therefore interfere with the inhibitory effect of the enzymatic activity [22]. However, there is controversy about these data, and other studies have identified lower levels of folate in carriers of the 1298C allele [26].

In a previous study by our group, a relationship was found between higher levels of total cholesterol and LDL cholesterol in the MTHFR hypermethylated samples of patients with DR [5]. The proposed mechanism for these findings is related to the reduction of MTHFR expression in the hypermethylated profile [18] that could result in higher concentrations of homocysteine, which in turn stimulates hepatic cholesterol synthesis [27].

In the present study, it was demonstrated that individuals with the hypermethylated profile and AA genotype of the A1298C polymorphism had higher levels of TC and LDL and also glycemia and HbA1C than did those with the genotype containing the C allele. Regarding glycemic control, evidenced through fasting glycemia and HbA1C analysis, the results were significantly higher in the AA group only in control group, whereas for the lipid parameters, the relationship occurred in both groups for total cholesterol and only in complication group for LDL cholesterol.

Haplotype analysis revealed that increased levels of total cholesterol and LDL were elevated in patients with a hypermethylated profile and 1298AA genotype independent of the C677T genotype, ruling out the possibility of the result being related to the haplotype or being a consequence of a cross-effect. On the other hand, the effect on glycemic control parameters was only observed in the 677CC/1298AA haplotype.

As demonstrated in this and other studies, the DNA methylation profile, whether global or in specific genes, seems to be related to the pathophysiology of diabetes and its chronic complications [28]. The most likely hypothesis, as previously described, is that hypermethylation reduces the production of messenger RNA of the *MTHFR* gene. At the same time, the level of MTHFR activity, mediated by the A1298C and C677T polymorphisms, may impact the metabolic pathway of the enzyme, affecting the formation and availability of SAM and consequently impacting the methylation profile of the carriers. However, the results of this study suggest that this appears to be true only when the promoter of the gene is hypermethylated, thereby reducing expression and strengthening the biological effect of the A1298C polymorphism. Surprisingly, no biologically important relationships were found in the analyses of the C677T polymorphism, which is precisely what has the most significant impacts on the enzymatic activity.

Both glycemic control and dyslipidemia are important biochemical factors related to diabetes complications. The results presented here demonstrate for the first time, to our knowledge, that the methylation profile associated with common genotypes of MTHFR are very significantly related to levels of HbA1C, glycemia, total cholesterol and LDL cholesterol. This work refines previously published data relating the hypermethylated profile to the occurrence of chronic complications in diabetes, especially diabetic retinopathy. In addition to genotypic distribution and biochemical analysis, considering the methylation profile and genotype, we can suggest that patients with genotype 1298AA and a hypermethylated profile present a worse metabolic situation.

Interestingly, epigenetic marker profiles are reversible. This has already been demonstrated in cultured human cells for the *MTHFR* gene [18]. Thus, studies such as these that show unfavorable metabolic conditions in certain profiles can define groups of patients who need observation and differential treatment, in addition to allowing the monitoring of the effectiveness of therapeutic interventions.

This study has some methodological weaknesses that need to be taken into account. Although the population analyzed was recruited on the basis of strict exclusion criteria, restricted to only patients with diabetes time between 5 and 10 years, the experimental number is small. The plasma homocysteine variable, not analyzed in this study, could help to confirm some assumptions made in the discussion of the results. The promoter methylation analysis technique does not assess the integrity of the CpG islands of the gene promoter. Finally, the absence of unmethylated samples in the studied sample impairs the understanding of the relationship between the methylation profile and the studied genotypes.

## Conclusion

The hypermethylated methylation profile associated with the 1298AA genotype appeared to be connected to higher values of glycemia, total cholesterol and LDL cholesterol.

## Abbreviations

AGP: alpha 1 acid glycoprotein
TAC: total antioxidant capacity
COL T: total cholesterol
CpG: cytosine/phosphodiester-linked guanine
CREA-S: serum creatinine
EDTA: ethylenediaminetetraacetic acid
BG: blood glucose
HbA1c: glycated hemoglobin
Hcy: homocysteine
HDL: high-density lipoprotein
LDL: low-density lipoprotein
M. ALB: microalbuminuria
MDA: malondialdehyde
MTHFR: 5,10-methylenetetrahydrofolate reductase
DN: diabetic nephropathy
CRP: C-reactive protein
DR: diabetic retinopathy
SAMe: *S*-adenosylmethionine
TRIG: triglycerides
